# Diagnostic Value of Spiral CT and Magnetic Resonance Imaging Scanning in Gastric Cancer and Precancerous Lesions

**DOI:** 10.1155/2022/3627385

**Published:** 2022-05-23

**Authors:** Yaolan Zhen, Qing Xie, Lei Liu

**Affiliations:** Oncology Department, Xianning Center Hospital, Xianning, Hubei 437100, China

## Abstract

In order to explore the diagnostic value of spiral CT and magnetic resonance imaging scanning in gastric cancer and precancerous lesions, the author selected 56 gastric cancer patients treated in a medical center (group) as the experimental subjects, and all patients underwent MRI, multislice spiral CT scan, and enhanced CT scan two weeks before surgery; at the same time, the gastric cancer staging results of patients were diagnosed according to surgical pathology. All patients were examined under the condition of knowledge and performed breath-holding exercise before examination. The status, location, and extent of tumor lesions were evaluated. In comparison of T staging of gastric cancer patients with magnetic resonance scanning imaging and postoperative pathological examination results, among them, T staging of 3 patients did not match the results of pathological examination, the accuracy rates of T staging on magnetic resonance scanning imaging were T1 = 94.7%, T2 = 87.6%, T3 = 91.2%, and T4 = 94.7%, and the total accuracy was 92.1%. Comparison of helical CT scan imaging and postoperative pathological examination results is as follows. Among them, T staging of 8 patients did not match the results of pathological examination, 3 patients were ulcerative, 5 were protuberance, the accuracy rates of T staging in spiral CT scan imaging were T1 = 90.8%, T2 = 82.2%, T3 = 76.9%, and T4 = 87.6%, and the total accuracy was 84.5%. The total accuracy rate of imaging N staging was 77.5%, and the total accuracy rate of spiral CT scanning imaging N staging was 80.8%. The accuracy rates of M0 and M1 staging in magnetic resonance imaging were 100.0% and 96.5%, respectively, and the accuracy rates of M0 and M1 staging in spiral CT scan imaging were 96.5% and 96.5%, respectively. The accuracy rate of magnetic resonance imaging for the diagnosis of gastric cancer N staging was 77.4%, and the reason for the low accuracy rate was mainly because the enhancement effect was not obvious due to insufficient enhancement. The accuracy rate of spiral CT in diagnosing N staging of gastric cancer was 80.9%, which was mainly due to the small diameter of the middle celiac artery lymph nodes. Magnetic resonance and spiral CT scans have high value in the early diagnosis and staging of gastric cancer.

## 1. Introduction

Gastric cancer is a common disease in oncology, and men over the age of 50 are the high-risk group. As a malignant tumor, the incidence of gastric cancer is extremely high, there are obvious regional differences, and the incidence of gastric cancer in the northern region is significantly higher than that in the southern region [1]. With the change of people's life and diet structure and the increasing pressure of life, the current incidence of gastric cancer is increasing year by year, and it is getting younger and younger. When the patient has onset, the early symptoms are not obvious, some patients are often accompanied by nausea, belching, abdominal discomfort, and other symptoms, and serious complications such as pathological tissue changes, upper gastrointestinal symptoms, melena, perforation of tumor ulcers, and jaundice may occur in patients with advanced disease. To this end, it should be detected and treated early [2]. The direction of preoperative evaluation of gastric cancer mainly includes lymph node metastasis and tumor invasion depth. With the development of imaging, a variety of imaging detection methods are used to evaluate the development of gastric cancer before surgery, including MRI, CT, EUS, B-ultrasound, gastroscope, and PET-CT Figure 1 shows the principle of MRI instrument [3]. Gastroscopy is mostly used for the qualitative diagnosis of gastric cancer and is the gold standard for preoperative diagnosis of gastric cancer; however, gastroscope cannot be used to evaluate lymph node metastasis and tumor invasion depth. B-ultrasound shows better sensitivity for diagnosing enlarged lymph nodes, but the disadvantage is that it is easily disturbed by abdominal gas or fluid; although to a certain extent, it can indicate the existence of lymphadenopathy, but it is impossible to make a qualitative diagnosis of lymph node metastasis, and B-ultrasound is rarely used to evaluate the stage of lymph node metastasis. Endoscopic ultrasonography shows good diagnostic value for the depth of tumor invasion and has good specificity for the diagnosis of lymph node metastasis but poor sensitivity; therefore, the diagnostic value of lymph node staging is poor. PET-CT has shown good diagnostic value for various tumors, but it is expensive and time-consuming; therefore, PET-CT is rarely used for preoperative evaluation in clinical practice. MRI scans, especially DWI imaging, show good specificity for the diagnosis of lymph node metastasis. Considering the evaluation value of gastric cancer, MRI is often used as an alternative to MDCT examination, and MRI is less directly used to assess the development of gastric cancer [4]. A number of previous studies have shown that MDCT has good sensitivity and specificity for evaluating lymph node metastasis, and it is also the most commonly used preoperative evaluation method in clinical practice.

## 2. Literature Review

In response to this research question, Gustinucci et al. stated that in the diagnosis of gastric cancer, research on the characteristics and accuracy of multislice spiral CT and 3.0 T magnetic resonance imaging provides a more reliable basis for the evaluation of subsequent clinical manifestations [5]. Bartpho et al. compared the value of multislice spiral CT and magnetic resonance imaging (MRI) in the diagnosis of gastric cancer N staging [6]. Zullo et al. stated that in the examination of primary gastric cancer lesions, CT and magnetic resonance imaging diagnostic methods can be used to detect lesions, a certain examination efficiency can be obtained, the application of the magnetic resonance examination method is as follows, the effect is more obvious, and the advantages are more significant; in the application of the corresponding spiral detection method for judgment, the corresponding treatment method can also be formulated through this effective treatment plan, in terms of its role. Its targeted use requirements also meet the actual use reference value [7]. Yi et al. showed that MRI is also more sensitive than CT imaging in detecting perineural spread and pathological lymph nodes [8]. He et al. showed that perineural dissemination and pathological lymph nodes were significantly associated with clinical treatment and prognosis [9]. Gopi et al. analyzed the MRI findings of 9 palatal tumors and found that MRI had significant advantages in assessing structures surrounding malignant tumor infiltration [10]. Aló et al. summarized the typical CT and MRI imaging findings of different histological types of palatal tumors and tumor-like lesions and found that conventional MRI signs can help narrow the range of differential diagnosis [11]. Cesare et al. studied the apparent diffusion coefficient (ADC) value of 32 salivary gland tumors (17 benign and 15 malignant) examined by preoperative diffusion-weighted imaging (DWI), they found that the ADC value could not reliably distinguish benign and malignant salivary gland tumors, and they speculated that the possible reason was that some salivary gland malignancies such as acinar cell carcinoma contained rich extracellular matrix, which led to the increase of the corresponding ADC value [12]. Simo et al. stated that retrospective imaging of 42 patients with parotid adenocarcinoma with conventional MRI and DWI showed that the sensitivity of DWI in the differential diagnosis of critical and benign disease with an ADC value of 1.02 × 10 − 3 mm^2^/s. Cancers were as follows: 87.5% and specificity 75.0%. Compared with conventional MRI, DWI was nontoxic and did not significantly improve the differential diagnosis of cancer, suggesting that conventional MRI remains the most valuable diagnostic tool for palate cancer [13]. On the basis of the current research, the author selected 56 gastric cancer patients treated in a medical center (group) as the experimental subjects, and all patients underwent MRI, multislice spiral CT scan, and enhanced CT scan two weeks before surgery; at the same time, the gastric cancer staging results of patients were diagnosed according to surgical pathology. All patients were examined under the condition of knowledge and performed breath-holding exercise before examination. The reason for the low accuracy rate is mainly because the enhancement is not enough; so, the effect after enhancement is not obvious: the accuracy rate of spiral CT in diagnosing N staging of gastric cancer was 80.9%, which was mainly due to the small diameter of the middle celiac artery lymph nodes.

## 3. Methods

### 3.1. General Information

Fifty-six gastric cancer patients were treated at the medical center (group). All patients were diagnosed with gastric cancer by gastroscopy, and all patients underwent surgery voluntarily [14]. Among the 56 gastric cancer patients, 36 were male and 20 were female; the age ranged from 45 to 68 years, with an average of (55.7 ± 4.2) years old. Among them, 12 cases were gastric corpus cancer, 18 gastric fundus and cardia cancers, 12 gastric body and gastric cardia cancers, 9 gastric antral hilum cancers, and 5 gastric antral hilum and gastric corpus cancers.

### 3.2. Methods

All patients underwent magnetic resonance imaging, multislice spiral CT scan, and enhanced CT scan two weeks before surgery; at the same time, the gastric cancer staging results of patients were diagnosed according to surgical pathology. Patients underwent informed examinations and performed breath-holding exercises before examinations [4, 15], using Philips GvmscanIntera1.5 T superconducting MR instrument and 4-channel and 8-channel body phased array coil. The sense technology was used to examine the patient, and the patient fasted for 8 hours and drank plenty of water (about 400 ml); before the examination, intramuscular injection of anisodamine (15 mg) and 250 ml of warm water were performed, the patient was lying down, an 8-channel imaging coil was selected for magnetic resonance imaging, and the coronal and transverse planes were mainly scanned. Accelerated dynamic acquisition enhanced scan of gastric volume, slice thickness 5 mm, and slice interval 1 mm. The patient was given an intravenous injection of 1.5 ml/s of 15 ml of meglumine spray, and all data were input to the ADW4.5 processing station for high-density and multiplanar projection imaging [2, 16]. The patient was scanned with a GE Lightspeed QX/ICT scanner, the tube voltage was 120 kV, the tube current was adjusted according to the actual situation of the test (250~300 mA), the layer thickness was 1.0 mm, the pitch was 3, and the scanning time was 8 ~ 10 s. Half an hour before the multispiral CT scan, 20 mg of intramuscular anisodamine hydrochloride muscles prevents the normal peristalsis of the gastrointestinal tract, and none of the patients had the stomach inflated through a gastric tube. Upload the data to the workstation and perform reconstruction analysis on the images. 3 radiologists with rich clinical experience above the deputy chief physician analyze the scan results, and the 3 radiologists jointly judge that the patient is gastric cancer [9].

### 3.3. Diagnostic Criteria

The status, location, and extent of tumor lesions were evaluated. The depth of invasion (T) is divided into four grades from T1 to T4: T1 means the lesion is not obvious or not detected, T2 means full-thickness gastric wall infiltration but no infiltration at the outer boundary, T3 means full-thickness gastric wall infiltration but irregular infiltration at the outer boundary, and T4 indicates that all surrounding organs are infiltrated [17, 18]. Lymph node metastasis (N) is divided into five criteria: Nx, NO, N1, N2, and N3: Nx means no evaluation, N0 means no obvious metastasis, N1 means 1 ~ 6 metastasis values, N2 means 7 ~ 15 metastasis values, and N3 means >15 transfer values. Distant metastasis (M) is divided into three criteria: Mx, M0, and M1. Mx means no metastasis: metastasis, M0 means 3 metastasis values, and M1 means >12 metastasis values [19].

## 4. Results and Analysis

### 4.1. Comparison of T Staging of Gastric Cancer Patient Comparison of Magnetic Resonance Imaging and Postoperative Pathological Examination Results

Among them, T staging of 3 patients did not match the results of pathological examination. The accuracy rates of T staging on magnetic resonance scanning imaging were T1 = 94.7%, T2 = 87.6%, T3 = 91.2%, and T4 = 94.7%, and the total accuracy was 92.1%, see Table 1.

Comparison of helical CT scan imaging and postoperative pathological examination results is as follows: among them, T staging of 8 patients did not match the results of pathological examination, 3 patients were ulcerative, 5 were protuberance, the accuracy rates of T staging in spiral CT scan imaging were T1 = 90.8%, T2 = 82.2%, T3 = 76.9%, T4 = 87.6%, and the total accuracy was 84.5%, see Table 2.

### 4.2. Comparison of N Staging of Gastric Cancer Patients with MRI Scan

The total accuracy rate of imaging N staging was 77.5%, and the total accuracy rate of spiral CT scanning imaging N staging was 80.8%, see Table 3.

### 4.3. Comparison of M Stage of Gastric Cancer Patients

The accuracy rates of M0 and M1 staging in magnetic resonance imaging were 100.0% and 96.5%, respectively, and the accuracy rates of M0 and M1 staging in spiral CT scan imaging were 96.5% and 96.5%, respectively, see Table 4 and Figures 2 and 3.

## 5. Discussion

Gastric cancer is a malignant tumor with a high incidence in the digestive system. Different infiltration depths seriously affect the therapeutic effect of gastric cancer. In the past, CT scan, fiberoptic gastroscope, and X-ray gastrointestinal gas barium double angiography were commonly used in the diagnosis of gastric cancer; however, due to its slow imaging speed and magnetic resonance imaging, it is easily affected by factors such as respiration and gastrointestinal motility and has not been used clinically [20, 21]. In this study, spiral CT combined with enhanced scanning can show the thickness of gastric wall and the depth of invasion in patients with gastric cancer, as well as the TNM staging of gastric cancer. There are many factors that affect the results of the gastric wall test, including differences in patients' own physical constitution, testing equipment, and contrast agents [22]. During the magnetic resonance imaging examination, the author found that the signal of T1-weighted imaging was equal and slightly higher, and the signal of T2-weighted imaging was slightly higher and higher; at the same time, the folds on the gastric mucosa could be seen. In the early stage of gastric cancer, the use of enhanced scanning can detect the extent of the patient's lesions and tumors, and the use of enhanced scanning in the delayed phase is beneficial for tumor staging and diagnosis. The reason for the low accuracy rate is mainly because the enhancement is not enough; so, the effect after enhancement is not obvious: the accuracy rate of spiral CT in diagnosing N staging of gastric cancer was 80.9%, which was mainly due to the small diameter of the middle celiac artery lymph nodes.

## 6. Conclusion

The authors proposed the diagnostic value of spiral CT and magnetic resonance imaging in gastric cancer and precancerous lesions and evaluated the early diagnosis and TNM staging of gastric cancer by observing spiral CT and magnetic resonance imaging. Early diagnosis of gastric cancer and assessment of TNM staging include gastric cancer, precancerous spiral CT, and magnetic resonance imaging. A total of 56 gastric cancer patients underwent multi-incision helical tomography and magnetic resonance imaging before surgery. The preoperative staging of gastric cancer patients was evaluated according to the scanning images, and the postoperative pathological results were analyzed. Results. Compared with surgical and pathological diagnosis, the accuracy of MRI T-phase was 92.1%, the total accuracy of spiral CT was 84.5%, the accuracy of N-phase MRI was 77.5%, the general accuracy of spiral CT was 80.8%, the accuracy rate of MRM in detecting gastric cancer was 100.0%, and the accuracy rate of multislot spiral CT was 96.5%. Conclusion. Magnetic resonance imaging and spiral tomography are of great significance in the diagnosis of gastric cancer. Cancer patient. Due to the small number of cases in this study, the results of this study are limited, and further analysis and discussion are needed.

## Figures and Tables

**Figure 1:** Principle of MRI instrument.

**Figure 2:** Comparison of the results of MRI and spiral CT in the diagnosis of gastric cancer M0 staging and pathological detection.

**Figure 3:** Comparison of the results of MRI and spiral CT in the diagnosis and pathology of gastric cancer M1 stage.

**Table 1:** Comparison of magnetic resonance scan imaging and postoperative pathological examination results.

Magnetic resonance imaging	Sensitivity	Specificity	Positive predictive rate	Negative predictive rate	Accuracy
T1	85.8	95.8	75.1	97.8	94.7
T2	83.4	88.1	45.6	97.9	87.6
T3	92.8	90.6	76.6	97.5	91.2
T4	91.8	95.6	84.7	97.8	94.7

**Table 2:** Comparison of helical CT scan imaging and postoperative pathological examination results.

Spiral CT imaging	Sensitivity	Specificity	Positive predictive rate	Negative predictive rate	Accuracy
T1	75.1	92.1	42.8	97.8	90.8
T2	80.1	82.72	50.1	95.1	82.2
T3	70.1	80.67	66.8	82.8	76.9
T4	83.4	88.75	66.8	95.2	87.6

**Table 3:** Comparison of the results of magnetic resonance and spiral CT in the diagnosis and pathological examination of N stage of gastric cancer.

Method	Staging	Sensitivity	Specificity	Positive predictive rate	Negative predictive rate	Accuracy
Magnetic resonance imaging	N0	69.3	90.8	69.3	90.8	85.8
	N1	61.6	73.4	66.8	68.9	67.8
	N2	46.8	90.3	63.7	80.5	78.7
Spiral CT imaging	N0	71.5	80.8	55.7	89.6	78.7
	N1	80.1	77.5	74.2	82.9	78.7
	N2	73.4	90.3	73.4	90.3	85.8

**Table 4:** Comparison of the results of magnetic resonance and spiral CT in the diagnosis of gastric cancer M staging and pathological detection.

Method	Staging	Sensitivity	Specificity	Positive predictive rate	Negative predictive rate	Accuracy
Magnetic resonance imaging	M0	100	100	100	100	100
	M1	80.1	98.1	80.1	98.1	96.5
Spiral CT imaging	M0	95.8	100	100	83.4	96.5
	M1	88.8	97.8	88.8	97.8	96.5

## Data Availability

The data used to support the findings of this study are available from the corresponding author upon request.

## References

[1] Sun J., Yue Y., Li R., Sun Q., Guan Q. (2021). Detection of hpv e6/e7 mrna in the diagnosis of cervical cancer and precancerous lesions after kidney transplantation. *American Journal of Translational Research*.

[2] Zhang C. X., Wu C. T., Xiao L., Tang S. H. (2021). The diagnostic and clinicopathological value of trefoil factor 3 in patients with gastric cancer: a systematic review and meta-analysis. *Biomarkers*.

[3] Rothman R. K., Weinreb J., Zucconi W., Malhotra A. (2020). Diagnostic value of ct of chest, abdomen, and pelvis in patients with solitary and multiple brain lesions. *American Journal of Roentgenology*.

[4] Zan X., Guo Q., Ji R., Chen Z., Zhou Y. (2020). Mo1068 screening biomarkers associated with gastric cancer and precancerous lesions in high-risk area: cross-sectional study based on population-cohort. *Gastroenterology*.

[5] Gustinucci D., Ciccocioppo L., Coppola L., Negri G., Giorgi-Rossi P. (2021). Multicentre evaluation of hepika test clinical accuracy in diagnosing hpv-induced cancer and precancerous lesions of the uterine cervix. *Diagnostics*.

[6] Bartpho T. S., Wattanawongdon W., Tongtawee T., Paoin C., Dechsukhum C. (2020). Precancerous gastric lesions with Helicobacter pylori vacA+/babA2+/oipA+ genotype increase the risk of gastric cancer. *BioMed Research International*.

[7] Zullo A., Rago A., Felici S., Licci S., Toritto T. (2020). Onset and progression of precancerous lesions on gastric mucosa of patients treated for gastric lymphoma. *Journal of gastrointestinal and liver diseases: JGLD*.

[8] Yi Y., Hu Z., Li R., Chen L., Liu W. (2021). Effectiveness of banxia xiexin decoction in the treatment of precancerous lesions: a protocol for systematic review and meta-analysis. *Medicine*.

[9] He X., Wang Y. (2020). Progress in research on relationship between gastric non-hp bacteria and gastric cancer and precancerous conditions. *Chinese Journal of Gastroenterology*.

[10] Gopi I., Maragathavalli G. (2021). Complete blood count as a pathological diagnostic marker in oral precancerous lesions and conditions. *Journal of Research in Medical and Dental Science*.

[11] Aló P. L., Cicciarelli M., De Felice F., Quintiliani C., Corsi A., Polimeni A. (2021). Immunohistochemical differences in squamous precancerous and cancerous lesions of the oral cavity and the larynx: preliminary data. *Applied Sciences*.

[12] Di Cesare T., D’Alatri L., Marchese M. R. (2020). The prevalence of signs and symptoms of laryngopharyngeal reflux and laryngeal precancerous lesions in urban taxi drivers. *European Archives of Oto-Rhino-Laryngology*.

[13] Simo R. T., Tchakounte C. K., Kamdje A., Sidje L., Telefo P. B. (2021). Cervical cancer awareness and detection of precancerous lesions at two district health centres in the west region of Cameroon. *Asian Pacific Journal of Cancer Care*.

[14] Gullo I., Grillo F., Mastracci L. (2020). Precancerous lesions of the stomach, gastric cancer and hereditary gastric cancer syndromes. *Pathologica*.

[15] Lu C. N., Wu J., She Q., Deng B., Ding Y. B. (2021). Application value of serum pepsinogen and gastrin-17 in screening gastric precancerous lesions. *World Chinese Journal of Digestology*.

[16] Titov S. E., Anishchenko V. V., Poloz T. L., Veryaskina Y. A., Ustinov S. N. (2020). Differential diagnostics of gastric cancer and precancerous changes of the gastric mucosa using analysis of expression of six micrornas. *Klinicheskaia Laboratornaia Diagnostika*.

[17] Wang X. T., Ji Z. Z., Han F., Lyu B. (2021). A comparative study of new gastric cancer screening scoring system and new abc method for screening gastric cancer and precancerous lesions. *Zhonghua nei ke za zhi*.

[18] Xu X., Li L., Sharma A. (2021). Controlling messy errors in virtual reconstruction of random sports image capture points for complex systems. *International journal of system assurance engineering and management*.

[19] Shriram S., Jaya J., Shankar S., Ajay P. (2021). Deep learning-based real-time AI virtual mouse system using computer vision to avoid COVID-19 spread. *Journal of Healthcare Engineering*.

[20] Xin L., Jianqi L., Jiayao C., Fangchuan Z., Chengyu M. (2021). Study on treatment of printing and dyeing waste gas in the atmosphere with Ce-Mn/GF catalyst. *Arabian Journal of sciences*.

[21] Huang R. (2015). Framework for a smart adult education environment. *World Transactions on Engineering and Technology Education*.

[22] Mosiychuk L. M., Kushnirenko I. V., Tatarchuk O. M., Konenko I. S., Petishko O. P. (2020). Особенности цитокинового баланса у пациентов с предраковыми состояниями желудка в зависимости от изменений в структуре щитовидной железы. *Gastroenterology*.

